RETRACTED

# TRIM25 blockade by RNA interference inhibited migration and invasion of gastric cancer cells through TGF-β signaling

**DOI:** 10.1038/srep19070

**Published:** 2016-01-12

**Authors:** Zhenya Zhu, Yong Wang, Chunhui Zhang, Shiyong Yu, Qi Zhu, Kun Hou, Bo Yan

**Affiliations:** 1 Department of General Surgery, Shanghai Pudong District People’s Hospital, Shanghai 201299, China; 2 Department of General Surgery, Punan Hospital, Pudong New District, Shanghai 200125, China

## Abstract

Tripartite Motif Containing 25 (TRIM25), a member of TRIM proteins, has been found abnormally expressed in cancers of female reproductive system. Here, TRIM25 was conspicuously expressed in human gastric cancer (GC) tissues in which its higher expression generally correlated with the poor prognosis of patients. Small interfering RNA (siRNA)-mediated knockdown of TRIM25 expression in MGC-803 and AGS cells had no effects on cell proliferation, whereas reduced cell migration and invasion. Gene set enrichment analysis on The Cancer Genome Atlas stomach adenocarcinoma (STAD) dataset revealed that several signaling pathways, including the migration, E-cadherin and transforming growth factor-β (TGF-β) pathways, were enriched in TRIM25 higher expression patients. Moreover, ectopic expression of TRIM25 in a GC cell line with lower expression of TRIM25 significantly promoted the migration and invasion. Further experiments with TGF-β inhibitor suggested that TRIM25 may exert its function through TGF-β pathway. In summary, our results indicate that TRIM25 acts as an oncogene in GC and thus presents a novel target for the detection and treatment of GC.

Globally, gastric cancer (GC) ranks the fourth most frequent diagnosed malignant disease and a leading cause of cancer death^1^. GC is diagnosed at late stage after distant metastases have already developed. Although significant progresses have been achieved in surgery, chemotherapy and radiotherapy for GC in recent years, GC remains a serious health problem with the five-year survival rate of only 20%^2^. Therefore, a thorough understanding of the molecular mechanisms underlying gastric carcinogenesis and identification of new therapeutic targets for GC are urgently needed.

Tripartite Motif Containing 25 (TRIM25, also known as estrogen-responsive finger protein (EFP)) is a member of TRIM proteins. TRIM25 contains a RING-finger domain, two B-box domains and a coiled-coil domain, and functions as an E3 ubiquitin ligase^3^. An estrogen-responsive element (ERE) has been identified at the 3′-untranslated region (UTR) of TRIM25 gene and its expression is induced by estrogen^4^. In recent years, TRIM25 has been found to be abnormally expressed in cancers of the female reproductive system. It was reported that TRIM25 was overexpressed in breast cancer^5^,^6^ and ovarian cancer^7^. While in endometrial carcinoma, TRIM25 expression was down-regulated^8^. TRIM25 is thought to target 14-3-3 σ, a cell cycle regulator, for proteolysis and promoted breast cancer growth^5^,^9^. Other members of TRIM proteins, including TRIM28^10^, TRIM29^11^ and TRIM31^12^,^13^, have been reported to be upregulated in GC. However, little is known about the expression and functions of TRIM25 in GC.

RETRACTED

In the current study, we showed that the expression level of TRIM25 mRNA was higher in GC tissues than in normal tissues. A high abundance of TRIM25 was closely related with poor overall survival of GC patients. We also showed that knockdown of TRIM25 had no effects on the proliferation of GC cells, but inhibited the migration and invasion of GC cells. The involved possible mechanism was also explored. Taken together, these results suggest that TRIM25 could regulate gastric carcinogenesis and may serve as a potential target for antineoplastic therapies.

## Results

### TRIM25 is frequently upregulated in GC tissues

Given the fact that several members of TRIM proteins were upregulated in GC, we re-analyzed RNA-seq data downloaded from The Cancer Genome Atlas website (TCGA) stomach adenocarcinoma (STAD) dataset and found that the TRIM25 level was higher in GC tissues than in normal tissue controls (P < 0.0001) (Fig. 1A). We then assessed the mRNA level of TRIM25 in 90 pairs of GC tissues and non-tumorous tissues by qRT-PCR analysis. The relative level of TRIM25 mRNA compared with GAPDH were calculated using ∆Ct method. As shown in Fig. 1B, a significantly increased level of TRIM25 was seen in GC tissues, compared with the levels detected in normal tissue controls (*P* < 0.0001).

Further, the median value of relative level of TRIM25 mRNA (0.759) was set as cut-off value and 90 patients were divided into low expression group and high expression group. To investigate the clinical outcome of GC subtype with low or high TRIM25 expression, Kaplan-Meier survival analysis was carried out. As shown in Fig. 1C, the survival time was significantly longer in patients with TRIM25-low expression than that in patients with TRIM25-high expression (*P* < 0.05). These results revealed that TRIM25 expression was up-regulated in GC tissues, which was closely related with poor overall survival of GC patients.

### Knockdown of TRIM25 in GC cells

To investigate TRIM25 function *in vitro*, we examined TRIM25 expression in 6 GC cell lines. As shown in Fig. 1D, MGC-803 and AGS, characterized with higher expression of TRIM25 in both mRNA and protein levels, were selected to study the function of TRIM25. Two siRNAs specific to TRIM25 (siTRIM25-1 and siTRIM25-2) and a negative control siRNA (siNC) were transfected into MGC-803 and AGS cells and the level of TRIM25 was subsequently determined by immunoblotting and qRT-PCR analysis. As shown in Fig. 2A,B, both siRNAs efficiently suppressed TRIM25 expression and siTRIM25-1 with a higher efficiency was chosen for further assays.

RETRACTED

### Effects of TRIM25 siRNA on the proliferation of GC cells

We then evaluated cell proliferation by CCK-8 assay. Intriguingly, siTRIM25-1-transfected cells had similar proliferation rate with siNC-transfected cells and wild-type control (WT) cells (Fig. 3A, *P* < 0.05), suggesting that TRIM25 had no effect on the proliferation of GC cells.

### Effects of TRIM25 siRNA on GC cell metastasis

To determine whether TRIM25 siRNA is capable of influencing tumor cell metastasis, cell migrated and invasive capability was determined in MGC-803 and AGS cells transfected with either siTRIM25-1 or siNC through transwell assays. Compared with control groups (WT and siNC), migration of MGC-803 and AGS cells was reduced by 47.0% and 39.0% separately following the transfection of TRIM25 siRNA (Fig. 3B). Similarly, TRIM25 siRNA transfected-cells displayed impeded invasion in both MGC-803 and AGS cells. The invasion decreased by 61.7% and 37.3%, respectively (Fig. 3C).

### Investigation of TRIM25-associated pathways in GC

To identify TRIM25-associated pathways in GC, gene set enrichment analysis (GESA) was carried out by using data from TCGA STAD dataset. As shown in Fig. 4A, the migration, E-cadherin and transforming growth factor (TGF)-β signaling pathways were closely related with TRIM25 expression.

Then, we analyzed the expression of the migration (matrix metalloproteinase [MMP]-2 and MMP-9), E-cadherin (E-cadherin, β-catenin and fibronectin 1 [FN1]) and TGF-β signaling (TGF-β1 and bone morphogenetic protein [BMP]-4) pathways-related protein in MGC-803 and AGS cells at 48 h after transfection of either siTRIM25 or siRNA control. As shown in Fig. 4B,C, TRIM25 siRNA treatment resulted in a notable decrease in the expression of MMP-2, MMP-9, β-catenin, FN1, TGF-β1 and BMP-4, and a significant increase in the expression of E-cadherin. These results further validated the GSEA data.

### TRIM25 on the regulation of TGF-β signaling

Considering that the inhibitory effects of TRIM25 siRNA on TGF-β1 expression, we supposed that it could suppress TGF-β signaling. Thus, we detected the phosphorylation of Smad2 and Smad4, downstream of TGF-β1 by immunoblotting at 6 h post transfection. As shown in Fig. 4D,E, transfection of TRIM25 siRNA in GC cells remarkably repressed the phosphorylation of Smad2 and Smad4.

RETRACTED

In order to further confirm the involvement of TGF-β signaling, MKN-28 cells with a lower expression of TRIM25 was overexpressed with TRIM25 and treated with TGF-β inhibitor (SB-431542, Fig. 5). Cell migration and invasion of GC cells was significantly promoted by ectopic expression of TRIM25, but remarkably inhibited by treated with TGF-β inhibitor. Additionally, the inhibitory effects of SB-431542 on cell migration and invasion of GC cells was impaired by ectopic expression of TRIM25. The expression of MMP-2 and MMP-9, as well as the phosphorylation of Smad2 and Smad4 was also detected by immunoblotting (Fig. 6). SB-431542 significantly inhibited the levels of MMP-2, MMP-9, p-Smad2 and p-Smad4, and such effects were weaken by TRIM25 overexpression. These data indicated that TRIM25 may promote cell migration and invasion partially by activating TGF-β pathway.

## Discussion

Although TRIM proteins have been recently studied in different types of malignancies^3^ and other members of TRIM proteins^10^,^11^,^12^,^13^ have been found overexpressed in GC, the knowledge of the aberrant expression and possible role of TRIM25 in GC is still lacking. Here, we showed that expression of TRIM25 was significantly increased in GC tissues compared with normal controls, which is consistent with the analysis of TCGA STAD dataset. Moreover, the upregulation of TRIM25 in GC was probably related to the prognosis of GC, which implied the possible clinical value of TRIM25 in GC (Fig. 1).

The previous studies revealed that knockdown of TRIM25 suppressed cell growth of lung cancer cells^14^ and breast cancer cells^9^. However, our data showed that reduced expression of TRIM25 had no effects on the proliferation of GC cells (Fig. 3A). These different results following knockdown of TRIM25 may due to different types of transfected cells. Consistent with previous findings from lung cancer^14^, we also found that TRIM25 could also remarkably inhibit the migration of GC cells (Fig. 3B). In addition, we showed that knockdown of TRIM25 in GC cells could notably decrease cell invasive ability (Fig. 3C). On the contrary, ectopic expression of TRIM25 in a GC cell line with lower expression of TRIM25 could notably induce cell migration and invasion (Fig. 5B,C). Thus, our data suggest that TRIM25 may be important in the development of GC.

Although the molecular mechanism governing the function of TRIM25 was not fully clear, GSEA analysis based on TCGA STAD dataset identified that several cancer-related networks, including migration, E-cadherin and TGF-β pathways, were positively correlated with TRIM25 expression (Fig. 4A). Compelling evidence indicates that cell migration and invasion are important for cancer initiation, progression, and metastasis^15^. Epithelial-mesenchymal transition (EMT) has been proposed as a critical step for the progression of primary tumors towards metastases^16^,^17^. E-cadherin is regarded as the main factor of EMT, thus contributing to the malignant progression of most epithelial tumors^16^,^17^. TGF-β signaling pathway is not only an important suppressor of epithelial cell proliferation, but also a key regulator for EMT^18^. Other TRIM proteins have been shown to regulate TGF-β signaling^19^,^20^. In the present study, the expression of the migration (MMP-2 and MMP-9), E-cadherin (E-cadherin, β-catenin and FN1) and TGF-β signaling (TGF-β1 and BMP-4, p-Smad2 and p-Smad4) pathways-related protein was affected by TRIM25 siRNA treatment (Fig. 4B,C). Further, the inhibitory effects of TGF-β inhibitor, SB431542 on cell migration and invasion in GC cells was impaired by TRIM25 overexpression (Fig. 5), which suggested TRIM25 might promote cell migration and invasion partially by activating TGF-β pathway. Our data suggested that the upregulated expression of TRIM25 will enhance EMT to facilitate the development of GC and invasive property. Further studies will be necessary to explore these possibilities.

RETRACTED

In conclusion, TRIM25 was overexpressed in GC, and aberrant expression of TRIM25 can affect migration and invasion of GC cells, probably through regulating TGF-β signaling and other critical target genes. Therefore, inhibitory strategy against TRIM25 might be a potential therapeutic strategy for GC.

## Materials and Methods

### Tissue specimens and cell lines

GC tissues and matched non-tumorous tissues were collected from patients who underwent surgery at Department of General Surgery, People’s Hospital, Pudong New District (Shanghai, China) between February 2007 and June 2009. The matched non-tumorous tissues were taken from at least 5 cm distance from the edge of tumor tissues. Overall survival (OS) was defined as the interval between the dates of surgery and death. The protocols used in the study were in accordance with the approved guidelines by the independent ethics committee, People’s Hospital, Pudong New District. Written informed consent was obtained from all patients.

GC cell lines, MKN-45, MGC-803, BGC-823, MKN-28, AGS and SGC-7901 cells were obtained from Cell bank, Chinese Academy of Sciences (Shanghai, China). Cells were maintained in Dulbecco’s modified Eagle’s medium (DMEM, Life Technologies, Grand Island, NY, USA), supplemented with 10% fetal bovine serum (HyClone, Logan, UT, USA), 100 mg/ml penicillin G and 50 μg/ml streptomycin, at 37 °C in 5% CO_2_.

RETRACTED

### Small interfering RNAs (siRNAs), plasmid and cell transfection

siRNAs targeting TRIM25 (siTRIM25-1, 5′-GGGAUGAGUUCGAGUUUCUUU-3′; siTRIM25-2, 5′-GGCUCAGAACACUUGAUAU-3′) and scramble siRNA (siNC) were purchased from Genepharm Technologies (Shanghai, China). Human TRIM25 CDNA was cloned into pcDNA3 expression vector (Invitrogen, Carlsbad, CA, USA) by Genewiz Company (Shanghai, China). pcDNA3 expression vector was used as a negative control (NC). All transfections were done by using Lipofectamine 2000 (Invitrogen) according to the manufacture’s protocol.

### RNA extraction, cDNA synthesis, and quantitative real-time PCR

Total RNA was isolated from tissue specimens or cells with the TRizol reagent (Invitrogen) and reverse transcribed to cDNA according to the manufacturer’s protocol (Fermentas, Hanover, MD, USA). Quantitative real-time PCR (qRT-PCR) was carried out by using an ABI 7300 real-time PCR machine (Applied Biosystems, Foster City, CA) and SYBR Green PCR kit (Thermo Fisher Scientific, Rockford, IL, USA). The relative expression of genes (TRIM25 and GAPDH) was calculated with the 2-(ΔCt) method. The primers used are listed here (TRIM25-forward, 5′-GTCTCTACCCAGAACAGTTTCC-3′; TRIM25-reverse, 5′-ATCCAACACAGGCTGATTCC-3′; GAPDH-forward, 5′-CACCCACTCCTCCACCTTTG-3′; GAPDH-reverse, 5′-CCACCACCCTGTTGCTGTAG -3′).

### Immunoblotting and antibodies

Cells were lysed in ice-cold RIPA lysis buffer (1% NP40, 0.5% Na-deoxycolic acid and 0.1% SDS in PBS) with fresh added Protease inhibitor (Sigma-Aldrich, St Louis, MO, USA). Whole cell lysates with equal amount of protein were separate by SDS-PAGE and transferred onto polyvinylidene difluoride membranes (Millipore, Bredford, MA, USA). Membranes were blocked with 5% skim milk and then incubated with primary antibodies at 4 °C overnight. Membranes were visualized using the appropriate secondary antibody at room temperature for 1 h followed by the enhanced chemiluminescence (ECL) system (Pierce, Rockford, IL, USA) according to the instructions of the manufacturer. The intensity of the immunoblotting signals was quantified by the densitometry with Image J software (NIH, USA). All experiments were repeated at least three times. Sources of primary antibodies were as follows: TRIM25, transforming growth factor (TGF)-β1, bone morphogenetic protein (BMP) -4, fibronectin 1 (FN1), matrix metalloproteinase (MMP)-2 and MMP-9, Abcam (Cambridge, MA, USA); E-cadherin, β-catenin, p-Smad2, p-Smad4, Smad2, Smad4 and GAPDH, Cell Signaling Technology (Danvers, MA, USA). Horseradish peroxidase-conjugated secondary antibodies were purchased from Beyotime (Shanghai, China).

### Cell growth assays

The MGC-803 and AGS cells were plated in 6-well plates, incubated for 24 h, and then transfected with siNC or siTRIM25-1. After 48 h, cells were seeded onto 96-well plates and cell proliferation was determined at 0, 24, 48 and 72 h by using CCK-8 (Dojindo Lab, Kumamoto, Japan). At indicated time points, cells were incubated in CCK-8 solution in normal culture medium for 1 h at 37 °C. The absorbance of each well was measured with a microplate reader set at 450 nM. All experiments were performed in triplicate.

RETRACTED

### Migration and invasion assay

MGC-803 and AGS cells on 12-well plates were transfected with siNC, siTRIM25-1, TRIM25 expression plasmid or control plasmid (NC). For migration assay, 48 h after transfection, 1 × 10^5^ cells in serum-free media were added to the upper chamber of transwell insert (8 m pore size; Corning Costar, New York, NY, USA). For invasion assay, cells were added to the upper chamber with Matrigel-coated membrane (BD Bioscience, Franklin Lakes, NJ, USA). For cells transfected with TRIM25 expression plasmid or NC, DMSO or 10 μM TGF-β inhibitor, SB431542 (Sigma-Aldrich), was added to the upper chamber as indicated. Medium containing 20% FBS were added to the lower chamber. After 24 h, cells that did not migrate or invade through the pores were completely removed by a cotton swab. Migrated or invaded cells were fixed with 4% paraformaldehyde, stained with 0.2% crystal violet, and counted under a microscope.

### Bioinformatics analysis

The gene expression data were obtained at The Cancer Genome Atlas website (TCGA, https://tcga-data.nci.nih.gov/tcga/) for stomach adenocarcinoma (STAD) projects. To explore the biological pathways involved in GC pathogenesis through TRIM25, a gene set enrichment analysis (GSEA) was performed as previously described^21^.

### Statistical analysis

Data from three independent experiments were presented as the mean ± standard deviation (SD). Two-tailed student’s *t*-test was used to calculate *P* value, and *P* < 0.05 was considered as statistically significant. Statistical analysis was carried out using GraphPad Prism (San Diego, CA, USA).

## Additional Information

**How to cite this article**: Zhenya, Z. *et al.* TRIM25 blockade by RNA interference inhibited migration and invasion of gastric cancer cells through TGF-β signaling. *Sci. Rep.* **6**, 19070; doi: 10.1038/srep19070 (2016).

## Figures and Tables

**Figure 1:** Overexpression of TRIM25 in GC. (**A**) The gene expression data RNA-Seq analysis of TRIM25 mRNA expression in GC tissues (n = 32) and normal tissues (n = 250). RNA-Seq analysis used data download from TCGA (*P* < 0.0001). (**B**) The mRNA level of TRIM25 in 90 pairs of GC and normal tissue was detected by qRT-PCR. TRIM25 mRNA was significantly overexpressed in GC tissues as compared with non-tumorous tissues (*P* < 0.0001). (**C**) Overall survival analysis showed that TRIM25 lower expression tumors have a better prognosis than TRIM25 higher expression tumors (*P* < 0.05). (**D**) Expression levels of TRIM25 were checked in a panel of 6 human GC cell lines using qRT-PCR method (left panel) and immunoblotting (middle and right panels). Representative immunoblotting (middle panel) and quantitative results (right panel) were shown (*P < 0.05, **P < 0.01, ***P < 0.001).

RETRACTED

**Figure 2:** TRIM25 expression was suppressed by siRNA transfection in GC cells. Expression of TRIM25 in MGC-803 (**A**) and AGS cells (**B**) was analyzed by qRT-PCR (left panel) and immunoblotting (middle and right panels). WT: wild type cells; siNC: scrambled siRNA-transfected cells; siTRIM25-1, siTRIM25-2: TRIM25-siRNA-1 or TRIM25-siRNA-2 transfected cells (*P < 0.05, **P < 0.01).

**Figure 3:** Reduced expression of TRIM25 suppressed the migration and invasion of GC cells. (**A**) Cell proliferation was detected in MGC-803 and AGS cells by CCK-8 assay. (**B**) Migration of MGC-803 and AGS cells treated with TRIM25 siRNA-1 or control siRNA was checked using no-matrigel coated transwell chamber. (**C**) Invasive ability of MGC-803 and AGS cells treated with TRIM25 siRNA-1 or control siRNA was assessed by using matrigel-coated transwell chamber. Scale bar: 100 μm. WT: wild type cells; siNC: scrambled siRNA-transfected cells; siTRIM25-1: TRIM25-siRNA-1-transfected cells (***P < 0.01).

**Figure 4:** TRIM25 expression affected migration, E-cadherin and TGF-β signaling pathways. (**A**) GSEA was performed using TCGA dataset. TRIM25-higher expression was closely related with migration, E-cadherin and TGF-β signaling pathways. (**B,C**) Expression of the above three pathway related gene was evaluated by immunoblotting in MGC-803 and AGS cells at 48 h after transfected with TRIM25 siRNA-1 or control siRNA. (**D,E**) Phosphorylation of Smad2 and Smad4 was evaluated at 6 h after transfection by immunoblotting. WT: wild type cells; siNC: scrambled siRNA-transfected cells; siTRIM25-1: TRIM25-siRNA-1-transfected cells (*P < 0.05, **P < 0.01, ***P < 0.001).

**Figure 5:** Ectopic expression of TRIM25 reversed the effects of TGF-β inhibitor on the migration and invasion of MKN-28 cells. (**A**) MKN-28 cells was transfected with control plasmid (NC) or expression plasmid encoding TRIM25. 48 h after transfection, expression of TRIM25 was analyzed by qRT-PCR and immunoblotting. (**B,C**) MKN-28 cells transfected with TRIM25 or NC, and migration and invasion assay were performed in a transwell chamber containing either DMSO or 10 μM TGF-β inhibitor, SB431542 (Sigma). Scale bar: 100 μm.

RETRACTED

**Figure 6:** Ectopic expression of TRIM25 reversed the effects of TGF-β inhibitor on TGF-β signaling. (**A**) Expression of MMP-2 and MMP-9 was evaluated by immunoblotting. (**B**) Phosphorylation of Smad2 and Smad4 was determined by immunoblotting (*P < 0.05, **P < 0.01, ***P < 0.001).
